# Influence of Case Management Model Combined with Continuous Nursing Care on Compliance Behavior and Adverse Emotions in Elderly Patients with Lung Cancer: A Prospective Single-Center Case-Control Study

This article has been retracted.

**DOI:** 10.1155/2022/2601852

**Published:** 2022-08-24

**Authors:** Aomei Li, Jie Gao, Juan Ni, Yuxin Che, Qing Zhang, Qian Hu, Jie Pan, YuXin Ge, Zhenzhu Cao, Juan Ni

**Affiliations:** ^1^Department of Radiotherapy, Nanjing Jinling Hospital, Nanjing University School of Medicine, Nanjing, 210002 Jiangsu Province, China; ^2^Department of Cadre Ward, Nanjing Jinling Hospital, Nanjing University School of Medicine, Nanjing, 210002 Jiangsu Province, China; ^3^Department of Nursing, Nanjing Jinling Hospital, Nanjing University School of Medicine, Nanjing, 210002 Jiangsu Province, China; ^4^Department of Respiratory and Critical Care Medicine, Nanjing Jinling Hospital, Nanjing University School of Medicine, Nanjing, 210002 Jiangsu Province, China

## Abstract

**Aims:**

To ask lots of questions about finding the truth about the influence of the case management model combined with continuous nursing care on following the law behavior and negative feelings of love, hate, fear, etc. in old patients with lung scale-like cell cancer.

**Materials and Methods:**

One hundred and forty-three elderly patients with squamous cell carcinoma of the lung were selected for this prospective study, 10 cases were shed due to epidemic and transfer, and finally 68 cases were in the control group and 65 cases in the observation group. The differences in anxiety and depression scores, quality of life, and compliance behavior between the two groups were observed and compared.

**Results:**

After nursing, the self-rating anxiety scale (SAS) and self-rating depression scale (SDS) of the observation group were lower than those of the control group, while the social support score was significantly higher than that of the control group. The scores of psychological behavior, exercise status, drug taking, and balanced diet of the two groups were significantly improved, and the observation group was significantly improved. The scores of medical compliance behavior in the observation group were significantly higher than those in the control group, and the mental vitality score, social interaction score, emotional restriction score, and mental status of the patients in the observation group were significantly higher than those in the control group, and the above statistics showed that the difference was statistically significant (*P* < 0.05).

**Conclusion:**

The use of a case management model combined with extended care significantly improved the compliance behavior and anxiety and depression of elderly patients with squamous cell carcinoma of the lung and improved the quality of life and social support.

## 1. Introduction

Lung scale-like cell cancer ranks first in the number of times something happens and death of harmful tumors in China. Now, China has become the world's largest lung scale-like cell cancer country, and the number of times something happens is still on the rise. Cancer is attracting more and more attention from the worldwide care system, and efforts are made to invest medical useful things/valuable supplies and actively plan cancer prevention and care-related success plans/ways of reaching goals. With the continuous development of medical technology and care methods, cancer has become a long-term care heavy load affecting patients, their families, and the whole community of people in the world. Even from the beginning of identification of a disease or problem, or its cause and treatment, the quality of life will be deeply affected as patients enter the medical care system. In the process of long-term treatment and nursing, patients not only need to face different physical discomforts caused by disease and treatment but also need to face the mental heavy load from themselves, their families, and community of people in the world. And with the continuous increase of patients' health knowing about something, their needs for the choice of treatment methods, information learning, mental support, and other aspects have slowly came out. Therefore, it has become an extremely important issue for the nursing community to make the best use of the limited medical supplies to meet the different needs of patients, so that they can get all the information and spiritual support they need within the limited time and space. Our research found that the development of case management model has become an inevitable trend in combination with diseases, patient needs, medical resources, and other aspects.

The case management model was first proposed by the case management community of people in the world of America (CMSA), and its core content is as follows: according to the humanistic and social attributes of each patient, clearly and sensibly select the different useful things and valuable supplies available, and put into use the case management model to meet the complete and thorough health needs of patients. The case management model refers to a method of providing a coordinated, arranged buying and selling for someone else model of services to patients through regular contact between managers and patients to provide big happening now care [1]. Continued care refers to the process from the patient's decision to be hospitalized, having surgery, and after waking up from drugs that cause numbness or unconsciousness to the patient's discharge. With the increasing health awareness of patients, their needs for the choice of treatment methods, information acquisition, and psychological support have gradually emerged [2]. However, there are few related studies on the effect of the combination of the two on following the law behavior and feeling of love, hate, guilt, etc. of old lung scale-like cell cancer. Based on this, the aim of our study was to investigate the effects of a case management model combined with extended care on compliance behavior and dysphoria in elderly patients with squamous cell carcinoma of the lung.

## 2. Material and Methods

### 2.1. Research Object

Before the experiment in this study, fully communicate with the patients, introduce the content and process of the experiment, related risks, and possible bad reactions, sign the based on knowledge and learning permission-related form after getting the patient's permission, and inform the patients of the test results in strict obedience of the experimental procedures. According to the needed things of event(s) or object(s) that prove something-based medicine and the study of what causes disease for the sample size, this study randomly included 143 patients. According to the random number rest grouping method, they were divided into the control group and the instance of watching, noticing, or making a statement group, and 10 cases dropped out due to the new crown widespread disease, hospital move from one place to another, etc. In the end, there were 68 cases in the control group and 65 cases in the instance of watching, noticing, or making a statement group. The female status and age of the patients in the two groups had no effect on this study.

### 2.2. Criteria

Inclusion criteria are as follows: (i) all elderly patients with lung cancer in this study met the diagnostic criteria for elderly lung cancer in the “Consensus on the Diagnosis and Treatment of Locally Advanced Non-Small Cell lung cancer” [3], 20-75 years old, with normal cognitive function; (ii) no metastasis, expected survival period ≥ 6 months, no mental illness or family history of mental illness, unconscious disturbance, no comprehension, memory, and orientation cognitive impairment; and (iii) all included patients obtained the informed consent, and liver, kidney, and bone marrow functions were normal.

Exclusion criteria are as follows: (i) those who have taken drugs that affect mood in the past 3 months and the patients have poor compliance or severe organ dysfunction and (ii) receive targeted drug therapy or chemotherapy, patients undergoing radiotherapy, biological immunization, and other treatments during the period, protective medical care, or those with cognitive impairment.

### 2.3. Nursing Intervention Methods

#### 2.3.1. Continuation of Care

In the control group, continuous nursing was used, that is (the creation of/the beginning of the existence of), medical records: the old patients with lung scale-like cell cancer were treated and discharged from the hospital, and the follow-up records were established. Family follow-up survey: family follow-up guidance for special old patients with lung scale-like cell cancer. It mainly includes two aspects: first, to understand the rehabilitation and change of the patient through continuous follow-up, and second, through the understanding of the disease changes and continuity of the patient after leaving the hospital rehabilitation health guidance. These old patients with lung scale-like cell cancer were followed up every 2-3 weeks by nurses, and the family members of the old patients with lung scale-like cell cancer were informed of the follow-up time in advance. During the follow-up process, it is necessary to patiently communicate with patients and their families, understand their voices, and give face-to-face guidance. If necessary, one or two patients with better (helping to fight disease) effects can be taken as role models, and they are encouraged to communicate with each other and learn from each other. Telephone follow-up: when the old patients with lung scale-like cell cancer are discharged from the hospital, register the mobile phone numbers of the old patients with lung scale-like cell cancer to make sure that the mobile phone numbers are very close to the truth or true number, and inform the department of the old patients with lung scale-like cell cancer. Telephone follow-up once a week, ask about the patient's recent drug use, understand the patient's bad drug reactions, mental status, and daily life, talk with the patient's family, and patiently ask the patient's actual situation. For old patients with lung scale-like cell cancer with poor (following the law/doing as you are told), nurses should instruct the old patients with lung scale-like cell cancer to take medicines on time, stress the results of not taking medicines on time, and require family members of old patients with lung scale-like cell cancer to supervise. For old patients with scale-like cell cancer of the lung, nurses should tell the old patients with scale-like cell cancer of the lung how to relax, take more rest, do more housework, and do more physical work.

#### 2.3.2. Case Management Model

The instance of watching, noticing, or making a statement group put into use the case management model on the basis of the control group, namely, case management: a management team composed of attending doctors, nurses, mental counselors, and family members of old patients with lung scale-like cell cancer. Through the (when something becomes well-known) of mental health knowledge and case management model training for old patients with lung scale-like cell cancer, it helps them to understand the condition, development, and recurrence of elderly lung cancer-like cell carcinoma and the importance of group treatment. The process of figuring out the worth, amount, or quality of something of the status of old patients with lung scale-like cell cancer includes risk test, money-based income, change to help someone place to live and sleep, status of old patients with lung scale-like cell cancer, and medical history. According to the process of figuring out the worth, amount, or quality of something and summary results, the problems existing in old patients with lung scale-like cell cancer are classified and sorted, from easy to very hard; to find out the advantages of old patients with lung scale-like cell cancer, tap their possible greatness or power, and then plan a case management plan. Doctors, nurses, and family members of old patients with scale-like cell cancer of the lung discussed together to carefully study the disease data of old patients with scale-like cell cancer of the lung and plan a case management model plan based on the questions raised. Regularly follow up old patients with scale-like cell cancer of the lung to figure out the worth, amount, or quality of the after an operation effect. For old patients with scale-like cell cancer of the lung who have not reached the target, ask the reasons, change to make better/change to fit new conditions the treatment plan appropriately according to the situation, and plan new treatments for unresolved or newly appearing problems plan. Medical-cooperative nursing: 10 nurses with 3 to 5 years of medicine-based work experience were selected to provide nursing care for old patients with lung scale-like cell cancer. The medical-cooperative nursing was performed twice a week for 60 minutes each time. The clearly stated/particular content is as follows: encourage old patients with lung scale-like cell cancer to speak out their current negative feelings of love, hate, fear, etc., and nurses carefully study the event and development of negative thoughts according to the patients' statements and guide the patients to permit the flow of mental counseling. Then tell the content of nursing care to the old patients with lung scale-like cell cancer, and point out the different from what is usually expected thinking in the thinking process of the old patients with lung scale-like cell cancer, so that the old patients with lung scale-like cell cancer at first understand that their negative thinking is caused by their own something that is different from what is usually expected caused by the way of thinking; it gives a reason to do something the old patients with lung scale-like cell cancer to carry out early and subject to change self-regulation and mental counseling according to the guidance of medical care. It enables old patients with lung scale-like cell cancer to record their negative feelings of love, hate, fear, etc. in the form of a diary and change to make better/change to fit new conditions (action that helps a bad situation plan in real time according to the features of old patients with lung scale-like cell cancer) to accomplish or gain with effort the best effect. The patients were followed up for 6 months according to the agreed reexamination date, and the last follow-up will win for patients less than 6 months. Establish a back and forth/equal between people trust relationship with patients, encourage patients to express their feelings, listen patiently, explain the safety and need of surgery, and improve patients' confidence in surgical treatment. Provide decorated with a personal touch health guidance, provide effective social support methods, enable patients to get as much help and support as possible from their family, friends, and fellow workers, and build the confidence and courage to overcome the disease.

### 2.4. Observation Indicators

Patients were figured out the worth, amount, or quality of for fear and stress and depression before and after nursing: the self-rating fear and stress scale (SAS) [4] score is greater than 50 showing fear and stress, and the higher the score, the worse the fear and stress. Self-rating depression scale (SDS) score is greater than 53, there is depression, and the higher the score, the worse the depression. For social support score (SSRS) [5], there are 10 items with a total score of 66 points. The higher the score, the higher the level of social support. The above scales are not affected by factors such as age, female status, and money-based status. All of the above scales were independent of age, gender, and economic status, and all of Cronbach's alpha values measured before use were 0.924. Medical compliance score [6] includes mental behavior score, exercise score, drug taking score, and eating lots of different healthy food score, each of which is scored from 0 to 45 points. The higher the score, the better the patient's medical following the doing as you are told behavior. Quality of life score includes mental energy score, social interaction score, emotional limitation score, and mental status score, each of which is scored from 0 to 100 points. The higher the score, the better the quality of life of the patient. The quality of life score is the simplest and most commonly used method to figure out the worth, amount, or quality of the quality of life of patients. It is easy for patients to understand and accept and has good reliability and something is truly what it claims to be. The measured Cronbach's alpha value is 0.962, with high sensitivity and convenient recording. For the quality of life, the Chinese version of the Quality of Survival Measurement Scale for Patients with Pulmonary Squamous Cell Carcinoma (FACTL-L, V4.0) [7] was used for assessment, including physical status, social status, emotional status, functional status, and additional components, with 5 dimensions and 36 entries; taking into account the traditional Chinese cultural background, the entry on sexual life in family status was removed, i.e., 35 entries with 0-4 points each. These five dimensions were scored directly from 0 to 4 for the positive entries and reversed for the negative entries, i.e., 4 points for those who filled in the first level, 3 points for those who filled in the second level, and so on, with the higher the score, the better the quality of survival. The test-retest reliability of the scale was 0.844, and Cronbach's a coefficient in this study was 0.862. The test will be completed within 30 minutes by the patient independently before and after nursing without being affected by any internal and external factors.

### 2.5. Statistical Analysis

The data in this study were calculated using Excel and reviewed by two physicians. The selected data conformed to the normal distribution, and the data were entered into the computer system by the first author and the corresponding author and checked. SPSS 25.0 was used for statistics, and all included data were tested for normality and were in line with normal distribution, and then, SPSS 25.0 was used for statistical processing of the data. One-way ANOVA was used for measurement data expressed as mean ± standard deviation (*x* ± *s*), and *χ*^2^ test was used for count data expressed as percentage (%). The differences were statistically significant at *P* <0.05.

## 3. Results

### 3.1. General Data Analysis

There was no significant difference between the two groups in gender, average age, average course of disease, body mass index, education level, and other general data by *t* test and chi-square test (*P* > 0.05). See Table 1.

### 3.2. Comparison of Anxiety, Depression, and Social Support Scores

Before nursing, there were no significant differences in anxiety, depression, and social support scores between the two groups. After nursing, the SAS and SDS of the observation group were lower than those of the control group, while the social support score was significantly higher than that of the control group, and the difference was statistically significant (*P* < 0.05). See Figure 1.

### 3.3. Comparison of Medical Compliance Behavior Scores

Before nursing, there was no significant difference in the scores of medical compliance behavior between the two groups. After nursing, the scores of psychological behavior, physical activity, drug taking, and balanced diet of the two groups of patients were significantly improved, and the medical compliance behavior score of the observation group was significantly higher than that of the control group, and statistics showed that the difference was statistically significant (*P* < 0.05). See Figure 2.

### 3.4. Quality of Life Score Comparison

Before nursing, there was no significant difference in the quality of life scores between the two groups (*P* > 0.05). After nursing, the mental vitality score, social interaction score, emotional restriction score, and mental state score of the observation group were significantly higher than those of the control group, and statistics showed that the difference was statistically significant (*P* < 0.05). See Figure 3.

### 3.5. Quality of Life

Two-way repeated measures ANOVA of FACTL-L scores at different time points in the two groups showed that the interaction effects between different time points, groups, and time points and groups were statistically significant (*P* < 0.05). The FACTL-L scores of the same groups at different time points were analyzed by one-way repeated measures analysis of variance. The results showed that the FACTL-L scores of the two groups of patients at 3 months and 6 months after nursing were significantly higher than those before nursing. L scores were significantly higher than 3 months of nursing, and the differences were statistically significant (*P* < 0.05). See Figure 4.

## 4. Discussion

Advances in medical technology and lung cancer have enabled some patients with lung scale-like cell cancer to be detected early. Especially, the moving ahead or up of slightly harmful chest-related surgery has given support for improving the treatment effect of patients with lung scale-like cell cancer. These (features/qualities/traits) decide/figure out lung scale-like cell cancer. Cancer patients require case management changed to fit their healing/repairing needs [8]. Therefore, case management is recommended in patients with lung scale-like cell cancer. Carrying out case management projects needs/demands more manpower, multi-(related to control or punishment) working together/team effort among doctors, nurses, laboratory departments, pharmacy departments, nutrition departments, communication and links with the community, improvement of hospital information systems, and even gradual establishment of a national brought together (as one) interconnected system. The information management (raised, flat supporting surface) system needs the support of the leaders to help increase/show in a good way and develop smoothly [9]. In this study, a team of nurses with rich medicine-based experience was selected from the ward, and case management was used after well-thought-out training and test/evaluation [10]. In the current situation of not having enough workers, money, time, etc. for brought together (as one) training and certification, only a few people have participated in clearly connected or related training, and only under their leadership can conditions be created to appropriately help increase/show in a good way the idea and model of case management [11]. For the promotion of case management, the current mainland system does not have the support of clearly connected or related policies, and hospital leaders lack understanding of its importance. In the trial and exploring things stage, the case managers trained and selected cannot be completely independent of the ward scheduling. Scheduling and giving-out nurse (workers in general/hiring, training, and firing department) is the basis for putting into use case management [12]. In the research process, case managers need to invest more personal time and energy to complete the patient follow-up and follow up, which increases the extra workload, so the training of case managers and the establishment of positions need to be supported in the system to have a better development [13].

For the case management model in this study, the communication between nurses and patients was strengthened and improves the patient experience, increasing patient motivation to actively participate in the process of treatment and care and to effectively help patients recover [14]. This study found that old patients with lung scale-like cell cancer almost never actively communicated with medical staff at first, but communicated with other patients through social software (in a carefully-planned way), hiding signs of sickness and mental needs to reduce the heavy load on family members, but missing active guidance from nurses. Communication between patients alone may lead to bad results [15, 16]. Through the correction of wrong thinking, emotional support, and nursing of bad behavior habits, patients can talk and listen to each other [17]. It greatly reduces the mental heavy load of patients, such as encouraging patients to get out of bed properly, listening to light music, muscle relaxation, and deep breathing training [18]. Fear and stress and depression are the two most common negative feelings of love, hate, fear, etc. in patients. Fear and stress is a kind of irritability caused by too many worry about the safety, future, and preplanned future of relatives or oneself [18]. Depression is a negative feeling of love, hate, guilt, etc. such as negative thinking, sadness, and hopelessness [19]. The case management model is an advanced nursing model that aims to improve patients' knowledge of old lung scale-like cell cancer and improve their life after discharge by putting into use effective health education for patients [20].

Clearly connected or related studies have shown that patients with lung scale-like cell cancer suffer from a variety of signs of sickness during using powerful drugs to help cure disease, including stomach- and intestine-related signs of sickness such as nausea and vomiting, emotional signs of sickness such as sadness and fear and stress, and general signs of sickness such as shortness of breath and tiredness, which bring a lot of negativity to patients' lives [21]. The results of this study showed that patients with lung scale-like cell cancer had lower scores on the functional scale before (using powerful drugs to help cure disease), but lower scores on the sign of sickness scale and clearly stated/particular signs of sickness, especially in difficulty breathing and inability to have a bowel movement. There are many factors affecting the quality of life of patients with lung scale-like cell cancer going through (using powerful drugs to help cure disease), such as age; whether someone is single, married, divorced, etc.; education level; male/female status; religious belief; and social support, among which (using powerful drugs to help cure disease) drugs themselves have the greatest hit/effect on the quality of life of patients [22]. In this study, the case management work model was applied to the management of patients with lung scale-like cell cancer going through (using powerful drugs to help cure disease), to understand the patient's service needs before (using powerful drugs to help cure disease), to plan a (designed for one person) treatment plan for the patient [23]. Also, ward visits, health lectures, group education, WeChat (being talked about a lot on TV, online, etc.), and other methods are used to carry out goal-oriented one-to-one targeted case management, including breathing [24]. It has a good effect on expanding the strength of the breathing and lung-related muscles and improving the following the law/doing as you are told of the lungs and small tube (from the mouth to the lungs), which in turn has a positive effect on improving the quality of life of the patients [25]. Some studies have shown that patients with lung scale-like cell cancer are much more depressed than ordinary people and have a heavier self-perceived heavy load, which seriously affects the treatment of the disease and the quality of life of patients [26]. Self-perceived heavy load includes patients' concerns about their need to depend on others for physical care, worry about the emotional hit/effect of their illness and death on their family members, and concerns about important role responsibilities and responsibilities that cannot be satisfied [27]. It has a significant bad effect on the patient's mental state, leading to a reduction in guilt, depression, distress, heavy load, and self-perception. The putting into use effect of case management nursing practice: the physical and mental and social functions and overall quality of life of patients with lung scale-like cell cancer decreased to different degrees during the whole process of treatment and healing [28]. Medical staff should plan an overall plan for medicine-based and home care based on the test/evaluation and statement about a possible future event results, which demands the support of medical staff, relatives, friends, and community of people in the world [29]. Help patients to treat the disease correctly, maintain a comfortable mood, and improve the quality of life of patients in the process of treatment and healing/repairing [30]. Case management can directly solve the discomfort of patients through direct nursing, health education, information support, and mental support and can provide continuous guidance and help for patients from many dimensions to help increase/show in a good way their self-change to make better/related to changing something [31]. The use of the case management care model in the using powerful drugs to help cure disease of patients with lung scale-like cell cancer has accomplished or gained with effort results. The research results show that the case management care model has positive effects on the care of patients with lung scale-like cell cancer treated with using powerful drugs to help cure disease and improves the patient's care happiness from meeting a need or reaching a goal and saves medical care cost. This model helps patients better and is worth advocating [32]. Case management can improve pain-related signs of sickness and fear and stress in patients with lung scale-like cell cancer, and case management should be actively carried out for patients with lung scale-like cell cancer pain. This study shows that the case management model makes happy by meeting a need or reaching a goal the patient's health knowledge, mental needs, and social support needs, improves the quality of life, and is worthy of active development [33].

There are certain limits in this study: before the start of the study, the project managers done intensive training and evaluation of the nurses participating in the study, but in the course of practice, when they faced patient discussions (with other people) and problems, they also interacted with other medical staff. In the process of communication between departments, there is still lack of confidence and doubt, resulting in poor communication. In response to this situation, the project team organizes nurses to manage and do work exchanges once a week and provides good enough information and communication skill support for case management nurses through group discussions and book-related understanding/explanation. Information support and mental support are the two major focuses of case management. Since each nurse's knowledge structure is different, the information output to the patient may also be different, and the patient's personality, expression ability, and desire are different, and the degree of emotional and mental problems exposed is also different. Therefore, how to secure sure of the information supported quality of being very close to the truth or true number and effectiveness of mental support are the keys to the effective putting into use of case management. Through working in a group to get ideas sessions, the people who work to find information discussed and summarized the most common problems of patients at each stage and continuously improved the original case management problem manual for patients with lung scale-like cell cancer for use by case management nurses in practice.

In conclusion, the use of a case management model combined with extended care significantly improved the compliance behavior and anxiety and depression of elderly patients with squamous cell carcinoma of the lung and improved the quality of life and social support, providing a reference and basis for the care of elderly patients with squamous cell carcinoma of the lung.

## Figures and Tables

**Figure 1:** Anxiety, depression, and social support scores. We used Excel to input all data. The scores of anxiety, depression, and social support were expressed as mean ± standard deviation. Independent sample *t* test was used. After nursing, the SAS (a) and SDS (b) of the observation group were lower than the comparison group, and the social support score (c) was significantly higher than the comparison group, statistical *P* < 0.05, with significance.

**Figure 2:** The scores of medical compliance behavior of the two groups of patients. We used Excel to input all data, and the scores of compliance behaviors were expressed as mean ± standard deviation, and independent sample *t* test was used. After the nursing, the scores of psychobehavior (a), exercise status (b), drug taking score (c), and balanced diet score (d) were significantly improved in the observation group. The medical compliance behavior score of the group was significantly higher than that of the control group, with a statistical *P* < 0.05, which was significant.

**Figure 3:** The quality of life scores of the two groups of patients. We used Excel to enter all data, and the scores for quality of life were expressed as mean ± standard deviation, using independent sample *t* test. After the nursing, the mental vitality score (a), social interaction score (b), emotional restriction score (c), and mental state score (d) of the observation group were significantly improved. It was significantly higher than the control group, with statistical *P* < 0.05, which was significant.

**Figure 4:** Quality of life. Two-way repeated measures ANOVA of FACTL-L scores at different time points in the two groups showed that the interaction effects between different time points, groups, and time points and groups were statistically significant (*P* < 0.05). The FACTL-L scores of the same groups at different time points were analyzed by one-way repeated measures analysis of variance. The results showed that the FACTL-L scores of the two groups of patients at 3 months and 6 months after nursing were significantly higher than those before nursing. L scores were significantly higher than 3 months of nursing, and the differences were statistically significant (*P* < 0.05).

**Table 1:** Comparison of general data between the two groups (*n* ($\bar{x}\pm s$)).

Group	Gender (men/women)	Average age (age)	Average disease duration (year)	Body mass index (kg/m^2^)	Education level		
					High school and below	Undergraduate	Master degree and above
Control group (68)	48/20	76.59 ± 8.32	12.82 ± 1.34	17.97 ± 3.50	18	35	15
Observation group (65)	47/18	76.62 ± 8.31	12.93 ± 1.29	17.95 ± 3.45	17	31	17
*χ* ^2^ */t*	0.048	-0.038	-0.482	0.033	0.002	0.190	0.305
*P*	0.826	0.951	0.631	0.974	0.967	0.663	0.581

## Data Availability

No data were used to support this study.
